The article "Prevention and Detection Research of Intelligent Sports Rehabilitation under the Background of Artificial Intelligence" was retracted in 2022. Reason: concerns about the peer review.

# Prevention and Detection Research of Intelligent Sports Rehabilitation under the Background of Artificial Intelligence

**DOI:** 10.1155/2022/3347166

**Published:** 2022-05-04

**Authors:** Qiong Huang, Fubin Wang

**Affiliations:** Military Science & Physical Education Department, Jiangxi Institute of Fashion Technology, Nanchang, 330201 Jiangxi, China

## Abstract

Artificial intelligence can bring convenience to human life. In the field of sports rehabilitation, the application of artificial intelligence is becoming more and more in-depth. This paper is aimed at studying the prevention and detection of sports rehabilitation in the context of artificial intelligence and proposing a compliance control method for lower limb rehabilitation robots based on artificial neural networks. In this paper, a double closed-loop control system is designed: the outer loop is an adaptive impedance control model based on sEMG feedback, and the purpose is to adjust the predicted desired joint trajectories. In the inner loop, a sliding mode iterative learning controller is designed to suppress periodic disturbance and abnormal jitter and achieve stable tracking of the target trajectory. Finally, the control method is simulated and verified by matlab/simulink, and a statistical experiment is done on the patient's recovery. The experimental results show that the use of artificial intelligence technology can effectively increase the sensitivity of the control system and improve the recovery rate of patients. Compared with the traditional sports rehabilitation control system, the sensitivity is increased by 22.7%, and the patient recovery rate is increased by 10.4%, which is of great significance in the field of sports rehabilitation.

## 1. Introduction

In real life, sports rehabilitation is not only for people with sports injuries; it can also help patients with musculoskeletal system injuries, patients after orthopaedic surgery, and even some subhealthy people. Sports rehabilitation is a branch of rehabilitation medicine, and its essence is the integration of “sports” and “medicine.” Sports rehabilitation is a multidisciplinary professional, including equipment rehabilitation therapy, manual rehabilitation therapy, and active exercise of patients to repair sports injuries. Traditional rehabilitation training mainly relies on the manual training of rehabilitation physicians. It not only has low rehabilitation efficiency but also is limited by the clinical experience of rehabilitation physicians in terms of training intensity, training effect, and patients' subjective emotions. Due to the lack of timely and clear understanding of the emotional state of stroke patients, it is easy to make patients feel disgusted in the overall rehabilitation treatment, which is even more unfavorable for rehabilitation treatment. This is also the drawback of traditional rehabilitation treatment.

AI is capable of developing artificially constructed human consciousness and thought patterns, and it can replace humans in some jobs. At present, many countries in the world, such as the United States, Japan, and Germany, use artificial intelligence technology to bring convenience to the field of human life. The development level of artificial intelligence also represents the development level of the country to a certain extent. The update and application of artificial intelligence science and technology have brought a profound impact on the development of people and society [1, 2]. Whether human beings will be replaced by machines, whether they will be enslaved by artificial intelligence, and how to reasonably respond to the challenges posed by artificial intelligence, we urgently need to respond. Therefore, studying the impact of artificial intelligence on human and social development can make artificial intelligence better serve the society and human beings. All social practice activities are dedicated to the achievement of people's practical goals. Therefore, studying the impact of artificial intelligence on human and social development is helpful for adhering to the principle of human subjectivity in social practice activities. On the other hand, it guides people to correctly view the social risks brought by artificial intelligence and make timely prevention. After years of development, artificial intelligence has achieved commercial and scale effects in medical, manufacturing, and other fields. For example, automatic identification of industrial robots.

This topic aims at the rehabilitation of limb motor function and extracts the features of motor imagery EEG signals. In-depth research on feature selection and the design and implementation of sports rehabilitation training system can lay a foundation for the application of sports rehabilitation training system. It not only has very important theoretical significance but also has very high application value.

## 2. Related Work

Choi et al.'s experiments show that older people are more convenient and effective in using smart healthcare [3]. To improve segmentation performance for noise-affected images, Memon and Lee propose a number of variants of the standard fuzzy *C*-means (FCM) clustering algorithm that incorporate local spatial neighborhood information into image segmentation [4]. She et al. proposed a new type of lower limb rehabilitation machine. It is asymmetrical from left to right, and the structure and load of the machine can be easily adjusted to suit the different demands on the lower extremities. They designed and built a single-leg half-model machine prototype and gave partial results of preliminary experiments [5]. Kim and Bae proposed a new type of intelligent wheelchair in-vehicle system. Its main purpose is to help the elderly and the disabled to carry out daily activities as much as possible and to minimize the degree of secondary disability [6].

Kosar et al. described a genetic algorithm- (GA-) based fuzzy proportional-integral-derivative (FPID) controller scheme for two spacecraft docking maneuvers [7]. Zou et al. introduced a parallel wire-driven lower limb rehabilitation robot. The robot has a modular design, reconfigurable, multimodel, and good human-machine compatibility. It has made great contributions to solving the related technical problems of lower limb rehabilitation robots in the aspects of configuration design, ergonomic compatibility, light weight, and multimodel rehabilitation [8]. The sports rehabilitation system based on artificial fish swarm intelligence algorithm has a positive impact on the recovery of motor function of disabled patients. In order to better apply the detection system to the clinical treatment of disabled patients, Chao et al. built a sports rehabilitation detection system based on artificial fish swarm intelligence algorithm. Then, they tested the running performance. The study found that the frequency of the eddy current signal obtained by this system is 118.60 Hz. It can effectively collect the weak signal of the sensor, and the limb control ability of disabled patients can be improved after using the system. Therefore, the sports rehabilitation detection system is beneficial to the recovery of motor function of disabled patients. Their research provides theoretical basis for the improvement of sports rehabilitation detection system [9]. Although these experts have built sports rehabilitation models of artificial intelligence algorithms, they are only in the theoretical stage and have not been able to make specific experiments to confirm the feasibility of the theory.

## 3. Movement Rehabilitation Control Method Based on Artificial Neural Network

### 3.1. Artificial Neural Network

The human brain is the most efficient intelligent system in the world. The brilliant achievements of human development depend on the information processing ability, information storage ability, and learning ability of the human brain. Scientists continue to study the human brain to simulate the structure and operation of the human brain, hoping to find out the mystery of the human brain. During this period, the most famous artificial neural network was born [10, 11].

Artificial neural network connects artificial neurons to each other according to certain connection rules. In the process of artificial neural network learning, the weights of interconnected neurons will change according to certain rules. Therefore, the nature of artificial neural network is determined by its network structure, that is, the way of interconnection and learning between neurons. That is, it is determined by the way the weights change.

#### 3.1.1. Neurons

The basic building block of the human brain and deep learning is the neuron [12]. Neurons in the human brain connect to other neurons through dendrites and axon terminals. Neurons receive signals from their artificial neurons, which are connected to their dendrites, mimicking neurons in the human brain. Although a variety of neural networks have been proposed to solve various problems, the basic unit of neurons that make up a neural network, the neuron, has a similar structure. The structure of the artificial neuron is shown in Figure 1.

Artificial neurons need data processing from input to output. b1~bn represent the input of the neuron, w1~wn are the weights of each synapse of the neuron, and *d* represents the bias of the neuron. Summation represents the processing function of the input signal, formula represents the activation function of the neuron, and output represents the output of the neuron. The main function of the artificial neuron is to process the input of the neuron through the processing function and then use the activation function to calculate the input processed by the processing function to obtain the output of the neuron [13]. In general, the processing function generally uses the sum function. There are many kinds of activation functions, and the common ones are as follows:

1. Sigmoid function: Sigmoid function for hidden layer neuron output. It is a monotonically increasing function, its advantage is that its value range is [0,1]; therefore, the function expression of Sigmoid is:

(1) $$\begin{array}{c} \text{Sigmoid}\left(i\right)=\frac{1}{1+e^{‐\text{i}}}. \end{array}$$

The derivative of the sigmoid function is:

(2) $$\begin{array}{c} {\text{Sigmoid}}^{\prime }\left(i\right)=\frac{e^{-i}}{{\left(1+e^{-i}\right)}^{2}}=\text{Sigmoid}\left(i\right)\left(1‐\text{Sigmoid}\left(i\right)\right). \end{array}$$

(2) tanh function: the tanh function is an improvement of the Sigmoid function. Compared with the Sigmoid function, the mean value of the tanh function is 0. And in practical applications, the tanh function has better performance than the Sigmoid function, and its function expression is:

(3) $$\begin{array}{c} \tanh\left(i\right)=2\text{Sigmoid}\left(i\right)-1=\frac{2}{1+e^{-i}}-1. \end{array}$$

(3) Relu function: Relu function is a widely used activation function in recent years, and its function expression is:

(4) $$\begin{array}{c} f\left(i\right)=\max\left(0,i\right). \end{array}$$

Compared with the Sigmoid function and the tanh function, the Relu function has the advantages of fast convergence when using the SGD algorithm and does not need to use the exponential function, so the calculation is simple [14]. However, when the Relu function is applied, if the learning rate is too large, the function value may drop to 0, resulting in the phenomenon of neuron failure. Therefore, when using the Relu function as the activation function, an appropriate learning rate should be selected.

(4) Leaky-Relu function: the Leaky-Relu function is to overcome the disadvantage that the Relu function may lead to the failure of neurons when it is used as an activation function. The expression of the Leaky-Relu function is as follows:

(5) $$\begin{array}{c} f\left(i\right)=\left\{\begin{array}{c} \beta i,i<0,\\ i,i\geq 0. \end{array}\right. \end{array}$$

*β* is a constant with a small value, so that the Leaky-Relu function retains the gradient when the function value is less than 0 without changing the data distribution, thereby avoiding the situation of neuron failure [15].

In addition, other commonly used activation functions are as follows: cosine (Cos) activation function, sine (Sinc) activation function, Sinusoid function, absolute function, and so on.

#### 3.1.2. Types of Artificial Neural Networks

Neural networks are formed by interconnecting neurons. According to the different connections between neurons, common artificial neural networks are divided into the following types: feedforward neural networks, feedback neural networks, self-organizing neural networks, etc. [16–19].

1. Feedforward neural network: the learning ability of the neural network composed of single-layer neurons is extremely limited, and it can only deal with and, or, nonlinearly separable problems. However, in applications, it is often necessary to deal with nonlinear separable problems. The emergence of feedforward neural network solves this problem. Feedforward neural network is generally composed of input layer, hidden layer, and output layer. The input layer accepts external input to the neural network, and does not process the input signal. After the output layer and the hidden layer process the input signal, the output layer outputs the processing result of the neural network. The neurons between the various layers of the feedforward neural network are connected to each other in a fully connected manner, and the neurons in the same layer are not connected to each other [20].  Figure 2 shows a feedforward neural network with 3 layers

(2) Self-organizing network is a kind of neural network that can map similar samples to adjacent output neurons. Self-organizing network adopts a kind of neural network of competitive learning strategy and adopts unsupervised learning method to train training samples. The self-organizing network realizes the mapping of high-dimensional input samples to low-dimensional space by mapping high-dimensional input data into two-dimensional output neurons. The output layer neurons of the self-organizing network are arranged in a two-dimensional manner, and each output layer neuron has a weight vector. When a training sample is input to the input layer, the distance between the training sample and each output layer neuron is calculated, and the neuron with the smallest distance is selected as the winning neuron [21]. Subsequently, neurons around the winning neuron adjust their weight vectors to reduce the distance from the training samples. The self-organizing network structure is shown in Figure 3

Artificial neural networks are mathematical models and algorithms that imitate human behavior.

### 3.2. Feature Extraction of Motor Imagery EEG Signal Based on LCD and CSP

ISC component satisfies:

(6) $$\begin{array}{c} {aA}_{h+1}+\left(1-a\right)X_{h+1}=0,a\in \left(0,1\right), \end{array}$$

where

(7) $$\begin{array}{c} A_{h+1}=X_{h}+\frac{f_{h+1}-f_{h}}{f_{h+2}-f_{h}}\left(X_{h+2}-X_{h}\right). \end{array}$$

In general [22], take *a* = 0.5; in this case, the *A*_*h*+1_/*X*_*h*+1_ = −1.

Calculate the value *A*_*h*+1_(*h* = 2, 3, ⋯, *N*) according to formula (7), and then, bring it into formula (8) to calculate the value of *L*_*h*_:

(8) $$\begin{array}{c} L_{h}={aA}_{h}+\left(1-a\right)X_{h},h=2,3,\cdots ,N-1. \end{array}$$

The values of *A*_*h*_ and *L*_*h*_ are from 2 to *N* − 1, and the EE values of the endpoints *L*_1_ and *L*_*N*_ need to be estimated. By continuation, the extreme points of the left and right ends are obtained, and then, *h* is equal to 0 and *N* − 1, respectively, and the values of *A*_1_, *A*_*N*_, *L*_1_, and *L*_*N*_ are obtained according to formula (7) and formula (8).

In order to obtain the baseline, namely *BL*_1_, all *L*_1_, *L*_2_, ⋯, *L*_*N*_ are fitted with cubic splines to form a smooth curve.

The baseline is separated by subtracting the baseline from the original signal, namely,

(9) $$\begin{array}{c} h_{1}\left(t\right)=x\left(t\right)-{BL}_{1}\left(t\right). \end{array}$$

If *h*_1_(*t*) satisfies conditions (1), (2), that is, an intrinsic scale component, output ISC_1_ = *h*_1_(*t*).

Otherwise, take *h*_1_(*t*) as the original signal data, repeat the process, then

(10) $$\begin{array}{c} h_{11}\left(t\right)=h_{1}\left(t\right)-{BL}_{11}\left(t\right). \end{array}$$

If *h*_11_(*t*) still does not meet the two conditions of ISC, repeat the steps (1), (2), (3), (4), (5), and cycle *k* times until *h*_1*n*_(*t*) meets the conditions of the ISC component, then *h*_1*n*_(*t*) is the first ISC component, denoted by ISC_1_ = *h*_1*k*_(*t*), formula (11) separates the components from the original data to obtain a new signal, namely,

(11) $$\begin{array}{c} u_{1}\left(t\right)=x\left(t\right)-{\text{ISC}}_{1}. \end{array}$$

Then, *u*_1_(*t*) is regarded as the original signal data, and the process is repeated to obtain the second component ISC_2_. Repeat the loop *n* times until *u*_*n*_ is a monotonic or constant function. Obtain the *n* components of ISC_1_, ISC_2_, ⋯, ISC_*n*_ and the trend terms *u*_*n*_(*t*), *u*_*n*_(*t*) = *u*_*n*−1_(*t*) − *ISC*_*n*_, so that *x*(*t*) can be decomposed into the sum of *n* ISC components and the residual term of a monotonic or constant function, that is:

(12) $$\begin{array}{c} x\left(t\right)=\overset{n}{\underset{p=1}{\sum }}{\text{ISC}}_{p}\left(t\right)+r_{n}\left(t\right). \end{array}$$

Among them, the standard deviation method (standard deviation, SD) is the ISC component termination criterion in this chapter, and *SD* is defined as:

(13) $$\begin{array}{c} \text{SD}=\overset{T}{\underset{t=0}{\sum }}\left[\frac{{\left|h_{ik}\left(t\right)-h_{i\left(k-1\right)}\left(t\right)\right|}^{2}}{h_{i\left(k-1\right)}^{2}\left(t\right)}\right]. \end{array}$$

In the formula, *T* is the length of time. Generally, if the value of SD is less than 0.5, the ideal ISC component can be obtained.

Since the LCD still has a certain time consumption, the three channels C3, C4, and C*z* that contribute the most to the classification are selected for LCD decomposition. The decomposition level of each channel is 3, so 9 ISC components can be obtained from one experimental data. Integrate the obtained 9 ISC components with the original 22-channel EEG signal to obtain 31-channel signal data. The Hjorth parameter [23] is extracted from the signal data of these 31 channels.

The Hjorth parameters are three parameters used to describe the characteristics of EEG signals. The Hjorth parameter contains the average power *m*_0_, the average frequency estimate *m*_1_, and the frequency bandwidth estimate *m*_2_. Since the EEG signal is a discrete sequence collected by a computer, it is represented by *σ*_0_ as the variance of the discrete sequence *X*, and *σ*_1_ and *σ*_2_ are represented as the variance of the first derivative and the variance of the second derivative of *X*, respectively; therefore:

(14) $$\begin{array}{c} m_{0}=\sigma_{0}^{2},\\ m_{1}=\frac{\sigma_{1}}{\sigma_{0}},\\ m_{2}=\sqrt{{\left(\frac{\sigma_{2}}{\sigma_{1}}\right)}^{2}-{\left(\frac{\sigma_{1}}{\sigma_{0}}\right)}^{2}}. \end{array}$$

After LCD processing the 22-channel EEG data, 9 ISC components can be obtained. It performs Hjorth feature extraction on these 31 signal data, extracts 3 features for each channel, and then obtains the time-frequency domain feature *F*_1_ = [*f*_11_, *f*_12_, ⋯, *f*_1*K*_] ∈ *R*^1×*KP*^; here, *K* = 93.

### 3.3. Control Method

In order to enable patients to recover their exercise ability better and faster, according to the guidance of the theory of rehabilitation medicine, when the muscle strength of the patient is almost zero in the early stage of rehabilitation, the robot will drive the patient to perform passive training at a certain speed. In the middle of the training, when the patient recovers part of the muscle strength, the robot will assist the patient to maintain a certain speed for assistive training. At the end of the training, the patient is actively training, and the machine does not provide assistance or resistance to increase muscle strength. Therefore, this paper designs three training methods: passive, assisted, and active [24].

Of the three training methods, passive training is relatively simple. The circular motion of the patient driven by the robot at a constant speed can be regarded as position control, with the desired rotational speed as the input. It is a single-input single-output position control system with the actual speed as the output. There are many control methods to achieve this, commonly used are PID control, feedforward plus PD control, and calculation torque method [25]. Their control block diagram is shown in Figure 4.

PID control is as shown in Figure 4. PID is the abbreviation of proportional, integral, and derivative. The difference between the expected value and the actual value is used as the input of the PID. After proportional, integral and differential operations, it acts on the rehabilitation robot, so that the position of the crank can follow the desired position.

In passive training mode, the rotation speed of the crank is used as the desired input value, and the patient or physician can set the desired rotation speed. After PID control, the actual speed of the crank fluctuates within the desired speed range, so theoretically, the patient can be driven for passive training [26].

PID control is relatively simple, mainly in the determination of PID parameters [27]. In addition to the PID control method for position control, feedforward plus PD feedback control (as shown in Figure 5) and calculated torque method (as shown in Figure 6) are commonly used. The dynamic model of a general *n*-degree-of-freedom manipulator is:

(15) $$\begin{array}{c} M\left(x\right)\ddot{x}+L\left(x,\dot{x}\right)+N\dot{x}+D\left(\dot{x}\right)+g\left(x\right)=\tau , \end{array}$$

where *x* is the joint angle vector; *τ* is the joint drive torque vector; *M*(*x*) is the coefficient of inertial force; $L\left(x,\dot{x}\right)$ is the centrifugal force and Coriolis force term; $N\dot{x}$ is the term of viscous friction; $D\left(\dot{x}\right)$ is the term of kinetic friction; and *g*(*x*) is the gravity term.

Formula (15) establishes the relationship between the joint driving force and the joint motion state. The desired motion state of the crank is input through the feedforward method, and the desired crank driving torque can be obtained by inverse dynamics calculation. Since the actual model is not completely consistent with the established dynamic model, there is an error between the obtained expected driving torque and the actual value. This error is eliminated by PD control, and the algorithm of feedforward + PD control is shown in

(16) $$\begin{array}{c} \tau =\tau_{d}-L_{v}\dot{\alpha }-L_{p}\alpha , \end{array}$$

where *τ*_*d*_ is the expected driving torque calculated by inverse dynamics; *α* is the difference between the actual angle of the crank joint and the expected angle; and *L*_*p*_, *L*_*v*_ are the coefficients of angle difference and speed difference, respectively.

The calculated torque method is similar to the feedforward + PD control algorithm, except that the PD feedback operation is performed before the inverse dynamics calculation. The algorithm of the calculated torque method is shown in

(17) $$\begin{array}{c} \tau =M\left(x\right)\cdot \left({\ddot{x}}_{d}-L_{v}\dot{\alpha }-L_{p}\alpha \right)+L\left(x,\dot{x}\right)+N\dot{x}+D\left(\dot{x}\right)+g\left(x\right), \end{array}$$

where *x* is the joint angle vector; *τ* is the joint drive torque vector; *V* is the coefficient of inertial force; $L\left(x,\dot{x}\right)$ is the centrifugal force and Coriolis force term; $N\dot{x}$ is the term of viscous friction; $D\left(\dot{x}\right)$ is the term of kinetic friction; *g*(*x*) is the gravity term; *α* is the difference between the actual angle of the crank joint and the expected angle; and *L*_*p*_, *L*_*v*_ are the coefficients of angle difference and speed difference, respectively.

The assisted and active training mode is the process in which the patient and the robot work together to help the patient carry out rehabilitation training. When it comes to human-computer interaction, the patient and the machine exchange energy. Compliant control is necessary to ensure patient safety. The compliance control can be classified into the category of force control, and the commonly used force control methods include impedance control, force-position hybrid control, adaptive control, and fuzzy control [28]. Impedance control is first and foremost one of the basic control methods to achieve flexible control. Impedance control is to adjust the target impedance of the end manipulator, so that the force and position between the manipulator and the environment satisfy a certain dynamic relationship. Impedance control is not simply to control position or control force but to incorporate force control and position control into the same system and to realize position control while realizing force control. Impedance control is to achieve the desired position of the environment while applying the desired force to the environment by adjusting the dynamic relationship of force and position between the operating arm and the environment. This dynamic relationship is called target impedance. Usually, the target impedance is represented by a mass-spring-damper system, that is, by a second-order linear differential formula:

(18) $$\begin{array}{c} M_{d}\left(\ddot{Y}-{\ddot{Y}}_{d}\right)+B_{d}\left(\dot{Y}-{\dot{Y}}_{d}\right)+L_{d}\left(Y-Y_{d}\right)=F_{d}-F_{e}, \end{array}$$

where *M*_*d*_, *B*_*d*_, *L*_*d*_ are the inertia matrix, damping matrix, and stiffness matrix; $Y_{d},{\dot{Y}}_{d},{\ddot{Y}}_{d}$ are the desired position, velocity, and acceleration of the robot end; $Y,\dot{Y},\ddot{Y}$ are the actual position, velocity, and acceleration of the robot end; and *F*_*d*_, *F*_*e*_ are the expected and actual forces between the robot end and the environment.

There are generally two ways to implement impedance control, one is force-based impedance control, and the other is position-based impedance control. Force-based impedance control is performed in the outer loop by detecting the position of the end of the manipulator, which calculates the theoretical actual contact force according to the robot dynamics model. It then achieves the desired position through an inner loop force controller, the control block diagram shown in Figure 7. Because the sensor detects the end position, force-based impedance control is suitable for low stiffness external environments. Position-based impedance control is performed in the outer loop by detecting the force between the manipulator and the environment. It then converts the force through the impedance parameter into a correction for position, velocity, or acceleration. The inner loop implements the position tracking function for the position controller, and the control block diagram is shown in Figure 8.

The impedance control algorithm adopted in this paper is the position-based impedance control, and an impedance control algorithm is designed [29]. The state of crank rotation is measured by the encoder, and the human-machine interaction torque can be obtained through the human-machine dynamic model. Then, the human-computer interaction torque is converted into the crank position correction amount through the impedance parameter, which is added to the desired position and realized by the inner loop position control. The inner loop position control algorithm in this paper is implemented by PID control, so the impedance control algorithm is shown in formula (19) and formula (20):

(19) $$\begin{array}{c} Y^{\prime }=L^{-1}\left\{\frac{\left[M\left(x\right)\ddot{x}+L\left(x,\dot{x}\right)+N\dot{x}+D\left(\dot{x}\right)+g\left(x\right)\right]\times 2}{l\times \left[M_{d}s^{2}+N_{d}s+L_{d}\right]}\right\}. \end{array}$$

In the formula, *Y*′ is the position correction amount of the outer ring; *L*^−1^ is the inverse Laplace transform; *l* is the crank length; and *M*_*d*_, *N*_*d*_, *L*_*d*_ are the impedance parameters.

(20) $$\begin{array}{c} \tau =k_{p}\left(Y^{\prime }+Y_{d}\right)+k_{i}\left(Y^{\prime }+Y_{d}\right)+k_{d}\left(Y^{\prime }+Y_{d}\right). \end{array}$$

In the formula, *Y*′ is the position correction amount of the outer ring; *Y*_*d*_ is the desired position value; and *k*_*p*_, *k*_*i*_, *k*_*d*_ are the PID parameters;

## 4. Sports Rehabilitation Experimental Design and Result Analysis

### 4.1. Experimental Analysis of EEG Data Processing

In the experiment, 5 Ag/AgCl electrodes were used to record the EEG signals on the scalp, and the distribution of all channels is shown in Figure 9.

The dataset includes four imaginary movements of the left hand, right hand, feet, and tongue. 6 subjects recorded EEG datasets on two different days. Each dataset consists of 6 separate data strings separated by a rest period. Each data string contains 48 experiments, 12 experiments for each type of imaginary movement. So a dataset has 288 experiments.

During the experiment, the subjects sat in front of the computer and conducted the experiment according to the computer prompts. An experiment lasts 14 seconds, and the experiment sequence is shown in Figure 10.

At *t* = 0, a circle is displayed on the black screen, and at the same time, a short sound will remind the subjects to start the experiment. At *t* = 3.75 s, there will be an arrow up, down, left, or right (corresponding to tongue, feet, left hand, and right hand, respectively) to prompt the subject's imagining task. At *t* = 6 s, the arrow disappears. There was no feedback during this process, and the subjects performed motor imagery until the cross disappeared at *t* = 10 s.

During the experiment, the electrode sampling rate was 250 hz, and the signal was processed with a band-pass filter of 0.5 hz-100 hz and a notch filter of 50 hz. The dataset for each subject can be divided into two parts, the dataset train and evaluation, which, respectively, include 288 experiments.

In order to remove the artifact interference and improve the signal-to-noise ratio of the signal, it is necessary to filter the EEG signal first before extracting features. In this chapter, according to the characteristics of ERD and ERS, the data in the dataset is filtered at 8-30 Hz to remove interference. According to the literature, the data of 2.5 s-3.5 s is selected for classification processing, and the signals before and after filtering are shown in Figure 11.

Aiming at the problem of large amount of calculation in LCD and high dimension after feature fusion, three channels C3, C4, and C*z* with the greatest contribution are selected from the five groups of signals. The LCD time-frequency decomposition is performed on it, and each channel is decomposed to obtain 3 ISC components, a total of 9 ISC components. According to the method, frequency domain features are extracted for these 9 ISC components.  Figure 12 shows the ISC component diagram of the EEG signal of the C3 channel after being decomposed by LCDF1 in an experiment.

The original 5 groups of EEG signals and 9 ISC components are integrated, and then, spatial features and time-frequency domain features are extracted for the integrated signals. Finally, the two feature vectors *F*1 and *F*2 are fused into feature *F*, which is sorted by MCFS and then input to the SDRA classifier for training and testing.

### 4.2. Hand Exercise Rehabilitation Experiment

The control strategy of the hand rehabilitation robot designed in this paper is based on active control, and the core of active control is impedance control. The control system recognizes the external input force of the system and outputs the desired motion position to the position controller via the variable impedance control system. The specific process is described in the third part. Now, through the hand rehabilitation platform, the control method of active motion is tested. In theory, the motion control trajectory output by the impedance system designed in this paper is less sensitive to external forces. It focuses more on following the given ideal training trajectory. In order to verify whether the designed variable impedance system can complete the designed trajectory following target, the experiment of the motor following the ideal trajectory is now carried out. In this experiment, the input value of the force sensor is set as a series of random numbers that are automatically generated by the program and vary within a given range. No graphic description is given here, the motor steering controller based on passive motion design is removed, and the output of the motor encoder is collected, as shown in Figure 13.

The experimental results show that the peak value of motor one is higher, and the average value of motor one is 22.7% higher than that of motor two, which indicates that the sensitivity of motor one under artificial intelligence intervention is higher than that of motor two. It can be seen that in terms of motor control, the rotation of the motor is composed of a continuous sinusoidal curve. It proves that the impedance control link of the designed active rehabilitation system can be learned through the fuzzy neural network. It adjusts the system impedance to achieve the goal of controlling the motion trajectory to follow the ideal trajectory.

### 4.3. Comparative Experiment of Artificial Intelligence Sports Rehabilitation and Traditional Sports Rehabilitation

In the experiment, training actions rated 1 to 5 were selected for testing. After calculation, the DTW distance and HD distance are obtained, respectively, and then, the confidence level assigned by the system (this paper sets DTW(0.60) : HD(0.40)), the algorithm fusion calculation is performed, and the comprehensive rating of action flow matching is obtained.  Table 1 shows the statistical results of five groups of randomly selected test data.

The experimental results show that the recovery rate of patients under artificial intelligence intervention has been significantly improved, which is 10.4% higher than that of traditional sports rehabilitation training.

## 5. Discussion

Although the control system has been verified by Matlab/Simulink simulation in this paper, and good static and dynamic characteristics have been obtained, there is still a lack of experimental data verification in the experiment of the stand-up exercise rehabilitation training process. Next, the control method will be verified by physical experiments, and further work will be done to realize the practical application of the control system faster.

In terms of rehabilitation training strategies, although a systematic rehabilitation model has been established, a lot of work is still needed in the construction of patient database software. And the database software construction work needs to be perfected through many experiments.

According to the traditional rehabilitation training evaluation method, in the final rehabilitation effect evaluation, the patient's physical feeling during the whole rehabilitation training process, that is, the degree of pain, should be considered.

## 6. Conclusion

Artificial intelligence technology has been gradually applied to the field of sports rehabilitation because of its imitation, realization, and expansion of human intelligence behavior characteristics. Through a preliminary summary of the application of artificial intelligence in sports rehabilitation scientific research, assessment technology, and treatment technology, the work ideas and scientific research innovation in the field of rehabilitation will be expanded. First, AI provides a better means for sports rehabilitation scientific research. Second, the application of AI makes rehabilitation assessment more intuitive and accurate. Third, the application of AI in sports rehabilitation technology liberates therapists and makes treatment easier. With the continuous improvement and maturity of artificial intelligence, the intelligent direction of sports rehabilitation will become a new development trend in the future.

## Figures and Tables

**Figure 1:** Structure diagram of artificial neuron.

**Figure 2:** Structure diagram of feedforward neural network.

**Figure 3:** Self-organizing network structure diagram.

**Figure 4:** PID control.

**Figure 5:** Feedforward + PD feedback control.

**Figure 6:** Calculated moment method.

**Figure 7:** Force-based impedance control.

**Figure 8:** Position-based impedance control.

**Figure 9:** Schematic diagram of electrode positions arranged according to the international 10-20 system standard.

**Figure 10:** Time paradigm of data acquisition experiment.

**Figure 11:** Images before and after filtering the EEG signal of C3 channel.

**Figure 12:** ISC component diagram of EEG signal of C3 channel after being decomposed by LCD.

**Figure 13:** Motor rotation angle experiment using fuzzy impedance control output.

**Table 1:** Statistical results of action flow matching test data.

Group	DWT algorithm		HD algorithm		Comprehensive rating
	Distance value	Rating	Distance value	Rating	
1	26.65	Level 1	0.0041	Level 1	Level 1
2	25.56	Level 2	0.0087	Level 2	Level 2
3	19.87	Level 3	0.0054	Level 3	Level 3
4	30.91	Level 4	0.0085	Level 3	Level 4
5	40.65	Level 5	0.0175	Level 4	Level 5

## Data Availability

The data that support the findings of this study are available from the corresponding author upon reasonable request.
